The article "Impact of NF-κB pathway on the intervertebral disc inflammation and degeneration induced by over‐mechanical stretching stress" was retracted in 2022. Reasons: duplicated images; unreliable data.

# Impact of NF-κB pathway on the intervertebral disc inflammation and degeneration induced by over‐mechanical stretching stress

**DOI:** 10.1186/s12950-021-00273-9

**Published:** 2021-02-02

**Authors:** Hui Xu, Guobao Qi, Kunpeng Li, Keshi Yang, Dawei Luo, Zhongxu Cai

**Affiliations:** 1 Department of Spinal Surgery, Liaocheng People’s Hospital, No. 67, Dongchang Xilu Road, 252000 Liaocheng, Shandong China; 2 Department of Spinal Surgery, Dongying People’s Hospital, No. 317, Nanyi Road, 257091 Dongying, Shandong China

**Keywords:** NF-κB, Intervertebral disc, Inflammation, Degeneration, Mechanical stretching stress

## Abstract

**Background:**

Intervertebral disk degeneration (IVDD) contributes to low back pain. Increased cell apoptosis and inflammation, decreased extracellular matrix are associated with IVDD. Nuclear factor-kappa B (NF-κB) signaling pathway and inflammatory cytokines are implicated in the pathophysiology of IVDD.

**Methods:**

In present study, we established a mechanical stretching stress-stimulated nucleus pulposus (NP) cell model. We knocked down NF-κB p65 by siRNA transfection to inhibit NF-κB and evaluated the effects of NF-κB inhibition on intervertebral disk degeneration. We applied the mechanical stretching stress on NP cells and inhibited NF-κB by siRNA, then evaluated the expression of inflammatory cytokines, matrix metalloproteinase (MMP), aggrecan, collagen II, and monitored viability and apoptosis of NP cells.

**Results:**

Mechanical stretching stress induced the expression of TNF-α, IL-1β, NF-κB, MMP-3 and MMP-13, while inhibited the production of aggrecan and collagen II in NP cells. Mechanical stretching stress decreased the cell viability and induced apoptosis in NP cells. Inhibition of NF-κB by siRNA suppressed the production of TNF-α, IL-1β, NF-κB, MMP-3 and MMP-13, while upregulated the expression of aggrecan and collagen II in NP cells.

**Conclusions:**

Inhibition of NF-κB by knocking down p65 suppressed over-mechanical stretching stress-induced cell apoptosis and promoted viability in NP cell. Inhibition of NF-κB suppressed inflammation and degeneration of NP cells in IVDD.

## Background

In western country, low back pain affects up to 50 % of the population and becomes one of the major health problems [1]. It is widely acknowledged that intervertebral disk degeneration (IVDD) is the master factor implicated in low back pain [2].

The intervertebral disks (IVD), which are composed of annulus fibrosus (AF), nucleus pulposus (NP) and cartilaginous endplates, lie between vertebral bodies and link them together [3]. The IVDD is a complex process in which multiple factors, including increased inflammation, excessive apoptosis, loss of extracellular matrix, and excessive mechanical stretch have been implicated [4]. The excessive mechanical strain could induce inflammatory cytokines production in NP cells [5]. Tumor necrosis factor alpha (TNF-α) is a key contributor to the IVDD by promoting matrix metalloproteinase (MMP) expression and extra cellular matrix degradation, amplifying inflammation, inducing cell apoptosis, and decreasing collagen II and aggrecan expression [6–9]. Interleukin 1 beta (IL-1β) has similar functions to TNF-α in IVDD [10]. TNF-α and IL-1β are mainly produced and secreted by immune cells, but they are also secreted by IVD cells [11]. The expression of TNF-α and IL-1β are remarkably increased in degenerated IVDs and the expression level is positively correlated with disc degeneration degree [11]. Anti-TNF-α and IL-1β therapies have been shown to alleviate disc degeneration.

Nuclear factor-kappa B (NF-κB) is transcriptional factor with multiple functions. NF-κB family comprises five members including p50, p52, p65 (Rel-A), c-Rel, and Rel-B proteins which form homo- or heterodimers for function. The most abundant form of NF-κB activated by pathologic stimuli via the canonical pathway is the p65:p50 heterodimer [12]. NF-κB has been shown to be critical in inflammation. Under unstimulated stage, NF-κB is inactive and present in cell cytosol. When stimulated by various stimuli including pathogen-associated molecular patterns (PAMPs), IL-1β, and TNF-α, NF-κB is translocated into host cell nucleus and activate gene transcription, which exacerbate the inflammation [13]. Mechanical stress can activate NF-κB signaling pathway and induce expression of TNF-α and IL-1β [14]. The significantly increased NF-κB activation is also identified in degenerated IVD tissues. Interestingly, inhibition of TNF-α, IL-1β or NF-κB by specific inhibitors or antagonists has been shown to ameliorate IVDD, suggesting these three factors are potential therapeutic target to treat IVDD [15–17]. SiRNA targeting NF-κB p65 has been shown to interfere the NF-κB signaling pathway and inhibit inflammation [18, 19]. In present study, using a mechanical stress-stimulated NP cell model, we inhibited NF-κB by siRNA treatment in NP cells and investigate the effects on IVDD.

## Materials and methods

### Nucleus Pulposus (NP) cell culture

NP cells were isolated from adult Sprague-Dwaley rats as described previously [20]. Briefly, the lumbar intervertebral discs were separated from the rats. Under a dissecting microscope, the gel-like nucleus pulposus were isolated and digested by 0.1 % collagenase II at 37°C for 6 h. The digested tissues were then transferred to DMEM/F12 medium containing 10 % fetal bovine serum and antibiotics (Thermo Fisher, Waltham, MA, USA). The cells were incubated at 37°C with 5 % CO_2_. Medium was changed every other day. The NP cells were harvested when was confluent.

The mechanical stretching stress was applied to the cells by using a four-point bending system (Mirui Technology Ltd, Chengdu, Sichuan, China) at the frequency of 1 Hz and different applied values (0, 1000 μ, 2000 μ, 4000 μ and 6000 μ) for 12 or 24 h. The general range of loading is from 100 to 6000 µ.

### Cell‐counting kit 8 (CCK-8) assay

NP cells were seeded in BioFlex® Culture Plates. After applying the stretching stress, the CCK-8 reagent (Abcam, Shanghai, China) for 3 h and the absorbance was read at 460 nm.

### Apoptosis assay

FITC Annexin V Apoptosis Detection Kit with PI kit (Biolegend, Beijing, China) was used to measure the apoptosis using flow cytometry. Briefly, NP cells were harvested and wash with FACS buffer (2 % fetal bovine serum in phosphate-buffered saline (PBS)). Cells were stained with the staining solution for 15 min at room temperature. After incubated with Annexin V binding buffer, cells were subjected to flow cytometry by using BD FACSCalibur Flow Cytometer.

### ELISA

Cell culture supernatants were collected after treatment. TNF-α and IL-1β were measured using commercial ELISA kits (Abcam, China) following manufacturer’s protocols.

### Western blot

Radioimmunoprecipitation lysis buffer (Abcam, China) was used for protein extraction. Extracted proteins were loaded on sodium dodecyl sulfate–polyacrylamide gel electrophoresis gel and then transferred to polyvinylidene fluoride membrane. After blocked with 5 % non-fat milk in PBST for 1 h at room temperature, membranes were incubated with primary antibodies for overnight at 4°C. Next day, after 3 times wash with PBST, corresponding secondary antibodies were incubated. The ECL Western Blotting Substrate (Abcam, China) was added to detect the reactive bands. The bands intensity was quantitated and analyzed by using ImageJ. The following primary antibodies were used: anti-NF-κB p65 (Abcam, China), anti-Bax (Abcam, China), anti-Bcl-2 (Abcam, China), anti-IL-1β (Abcam, China), anti-IL-6 (Abcam, China), anti-GAPDH (Abcam, China).

### RT-PCR

Total RNA was extracted using RNeasy Mini Kit (Qiagen China, Shanghai, China). The cDNA was synthesized and subjected to Real-time PCR by using QuantStudio 3 (Thermo Fisher, USA) and TB Green® Advantage® qPCR Premix (Takara, China). Primers used for RT-PCR were: p65 Forward: 5’-GAGACCTGGAGCAAGCCATT − 3’, Reverse: 5’-GCCTGGTCCCGTGAAATACA-3’. MMP-3 Forward: 5’- TTGATGGG CCT GGAATGGTC-3’, Reverse: 5’- AACAAGACTTCTCCCCGCAG − 3’. MMP-13 Forward: 5’-AAGCACCCCAAAACACCAGA-3’, Reverse: 5’-ACATGAGGTCTCGGGATGGA-3’. Aggrecan Forward: 5’-TCACCACCCACTCCGAAGAAGTTT-3’, Reverse: 5’-TCACCACCCA CTCCGAAGAAGTTT-3’. Collagen II Forward: 5’-CTCCATGTTGCAGAAGACTTTCA-3’, Reverse: 5’-TTCATGCATCCGCTAGTCCCTTCT-3’. TNF-α Forward: 5’-CCCTGGTACT AACTCCCAGAAA-3’, Reverse: 5’-TGTATGAGAGGGACGGAACC-3’. IL-1β Forward: 5’-C CAGGATGAGGACCCAAGCA − 3’, Reverse: 5’-TCCCGACCATTGCTGTTTCC-3’. β-actin Forward: 5’-CGTGCGTGACATCAAAGAGAAG-3’, Reverse 5’-CGTTGCCAATAGTGATGA CCTG-3’.

### SiRNA and transfection

The siRNA duplexes were designed by using Stealth RNAi Pre-Designed siRNAs online software (http://www.thermofisher.com/cn/zh/home/life-science/rnai/synthetic-rnai-analysis/stealth-select-rnai.html) and synthesized by GenePharma (GenePharma Co., Suzhou, China). The p65 siRNA duplexes sequences were: Sense 5’- GCAUGCGAUUCCGCUAUAAT T-3’, Antisense 5’- UUAUAGCGGAAUCGCAUGCTT − 3’. The control siRNA sequence were : Sense 5’- UUCUCCGAACGUGUCACGUTT-3’,Antisense 5’-ACGUGACACGUUCG GAGAATT-3’. Lipofectamine RNAiMAX (Thermo Fisher, USA) was used to transfect siRNA to NP cells following manufacturer’s instructions.

### Immunofluorescence assay

Cells were fixed with 4 % paraformaldehyde in PBS and permeabilized with 0.1 % Triton-X100. After blocking, anti-p65 antibody was added and incubated for 1 h at 37°C. After wash, cells were incubated with Alexa Fluor 488 conjugated secondary antibody and DAPI, and then mounted with ProLong™ Gold Antifade Mountant (Thermo Fisher, USA). Images were taken by Nikon ECLIPSE 80 i microscope.

### Statistical analysis

Experiments were independently repeated in triplicate. One- or two-way ANOVA analysis followed with an appropriate post hoc test was used to determine statistical difference. Statistical difference was considered as significant when *p* < 0.05.

## Results

### Mechanical stretching stress induced inflammation and degeneration in rat nucleus pulposus cells

To evaluate the effects of mechanical stretching stress on NP cells, we stretched NP cells with different values (0-6000µ) for 12 or 24 h, and monitored the cell viability, the production of TNF-α, an inflammatory cytokine associated with intervertebral disc degeneration, the expression of NP cells marker aggrecan and disc degenerative marker MMP-3. As shown in Fig. 1a and 1000 µ stretching for 12 or 24 h significantly increased the viability of NP cell. Increased stretching intensity resulted in decreased cell viability as 2000, 4000 and 6000 µ stretching for 12 or 24 h significantly reduced cell viability when compared to no stretching. 1000 µ stretching did not induced NP cells to produce TNF-α (Fig. 1b). In contrast, 2000, 4000 and 6000 µ stretching for 12 or 24 h resulted in significantly increased production of TNF-α in an intense-dependent manner. The highest value stretching (6000 µ) resulted in highest production of TNF-α. 1000 µ stretching significantly increased the mRNA level of aggrecan while intensified stretching resulted in significantly decreased mRNA level of aggrecan (Fig. 1c), which was in an intense-dependent manner. 1000 µ stretching did not affect mRNA level of MMP-3 while 2000, 4000 and 6000 µ stretching significantly increased the mRNA level of MMP-3 in an intense-dependent manner (Fig. 1d). Taken together, our data demonstrated that mechanical stretching decreased NP cell viability and expression of aggrecan while increased the expression of TNF-α and MMP-3, two factors associated with intervertebral disc degeneration. These results indicated that mechanical stretching stress induced inflammation and degeneration in NP cells. As 4000 µ stretching for 24 h gave the satisfied result, we adopted this condition for other studies.

**Fig. 1:** Mechanical stretching stress induced intervertebral disc inflammation and degeneration in rat nucleus pulposus cells. The cells in different groups were stretched mechanically by 1000µ, 2000µ, 4000µ and 6000µ respectively for 12 h and 24 h. CCK-8 was used to measure the cell viability (**a**), ELISA was used to measure the level of TNF-α (**b**), Real-time PCR was used to measure the mRNA expressions of Aggrecan (**c**) and MMP-3. Data are presented as mean ± SD. *p < 0.05, **p < 0.01, ***p < 0.001 compared to control

### SiRNA treatment prevented mechanical stretching stress induced NF-κB p65 expression

NF-κB signaling pathway can be activated by mechanical stress and played essential role in intervertebral disc degeneration [14, 21]. We transfected NP cells with NF-κB p65 siRNA and evaluated the effects on p65 expression after mechanical stretching stress stimulation. As shown in Fig. 2a&b, mechanical stretching stress significantly enhanced the expression of p65 in NP cells. Transfection of control siRNA to NP cells (si-NC group) did not affect the stretching stress-induced p65 expression. In contrast, transfection of siRNA against p65 significantly decreased the p65 level in NP cells after stretching stress stimulation. Similarly, transfection of p65 siRNA significantly reduced mRNA expression of p65 (Fig. 2d). Moreover, stretching stress stimulation induced NF-κB nuclear translocation. In contrast, in p65 siRNA transfected NP cells, there was no obvious nuclear translocation of p65 detected after stretching stress stimulation (Fig. 2c). Collectively, our data demonstrated that transfection of p65 siRNA knocked down endogenous p65 protein level and prevented mechanical stretching stress induced NF-κB p65 expression.

**Fig. 2:** Effects of NF-κB inhibition on over-mechanical stretching stress-induced p65 expression in rat nucleus pulposus cells. **a** Western blot analysis for the protein expression of p65, GAPDH was used as loading control. The relative expressions were normalized to control (**b**). **c** The nuclear translocation of p65 was measured by Fluorescence immunocytochemistry. **d** Real-time PCR was used to measure the mRNA expressions of p65. Data are presented as mean ± SD. ***p < 0.001 between the indicated groups

### Inhibition of NF-κB prevented mechanical stretching stress‐induced apoptosis of rat nucleus pulposus cells

We continued to evaluate the effects of NF-κB inhibition on stretching stress-induced cell death. Stretching stress stimulation significantly decreased cell viability in NP cells (Fig. 3a). In contrast, transfection of p65 siRNA significantly enhanced the cell viability in stretching stress-stimulated NP cells. The decreased cell viability after stretching stress stimulation was correlated to the enhanced apoptosis of NP cells (Fig. 3b&c). Knocking down p65 significantly reduced the stretching stress-induced apoptosis of NP cells (Fig. 3b&c). Correspondingly, stretching stress stimulation remarkably increased the Bax expression and decreased Bcl-2 expression (Fig. 3d&e). Knocking down p65 suppressed the expression of Bax while rescued Bcl-2 expression in stretching stress-stimulated NP cells. After quantitation, stretching stress significantly increased Bax/Bcl-2 ratio while knocking down p65 by siRNA transfection significantly decreased the Bax/Bcl-2 ratio in stretching stress-stimulated NP cells. Together, our data demonstrated that inhibition of NF-κB prevented stretching stress-induced apoptosis in NP cells.

**Fig. 3:** Effects of NF-κB inhibition on over-mechanical stretching stress induced apoptosis of rat nucleus pulposus cells. CCK-8 was used to measure the cell viability (**a**). Apoptotic cells were stained with Annexin V-PE and PI, and analyzed by flow cytometry (**b** and **c**). **d** Western blot analysis for the protein expression of Bax and Bcl-2. GAPDH was used as loading control. The relative expressions of Bax/Bco-2 were calculated (e). Data are presented as mean ± SD. *p < 0.05, **p < 0.01, ***p < 0.001 between the indicated groups

### Inhibition of NF-κB ameliorated mechanical stretching stress‐induced intervertebral disc degeneration in NP cells

Next, we investigated the effects of NF-κB inhibition on intervertebral disc degeneration by monitoring the expression of cell markers. Mechanical stretching stress significantly promoted the mRNA level of MMP-3 (Fig. 4a) and MMP-13 (Fig. 4b), two disc degeneration marker. In contrast, mechanical stretching stress significantly decreased the mRNA level of aggrecan (Fig. 4c) and collagen II (Fig. 4d). Transfection of p65 siRNA significantly decreased MMP-3 and MMP-13 mRNA level while rescued the mRNA expression of aggrecan and collagen II in mechanical stretching stress-stimulated NP cells. Collectively, our data demonstrated that inhibition of NF-κB p65 ameliorated mechanical stretching stress-induced degeneration in NP cells.

**Fig. 4:** Effects of NF-κB inhibition on over-mechanical stretching stress induced intervertebral disc degeneration in rat nucleus pulposus cells. Real-time PCR was used to measure the mRNA expressions of MMP-3 (**a**), MMP-13 (**b**), Aggrecan (**c**) and Collagen II (**d**). Data are presented as mean ± SD. *p < 0.05, **p < 0.01, ***p < 0.001 between the indicated groups

### Inhibition of NF-κB prevented mechanical stretching stress‐induced inflammation in NP cells

Lastly, we detected the effects of NF-κB inhibition on inflammatory cytokine production after mechanical stretching stress stimulation. We detected significantly increased TNF-α (Fig. 5a) and IL-1β (Fig. 5b) in NP cell culture supernatant after mechanical stretching stress stimulation. Inhibition of NF-κB by transfection of p65 siRNA significantly reduced both TNF-α and IL-1β production in mechanical stretching stress-stimulated NP cells. Correspondingly, we detected significantly increased mRNA level of TNF-α (Fig. 5c) and IL-1β (Fig. 5d) in mechanical stretching stress-stimulated NP cells while knocking down NF-κB p65 significantly decreased mRNA level of TNF-α (Fig. 5c&d) and IL-1β (Fig. 5d&f) in mechanical stretching stress-stimulated NP cells. Consistently, we detected remarkably increased TNF-α and IL-1β proteins in mechanical stretching stress-stimulated NP cells while knocking down NF-κB p65 decreased the protein level of TNF-α and IL-1β (Fig. 5d, e).

**Fig. 5:** Effects of NF-κB inhibition on over-mechanical stretching stress induced inflammation in rat nucleus pulposus cells. ELISA was used to measure the levels of TNF-α (**a**) and IL-1β (**b**). Real-time PCR was used to measure the mRNA expressions of TNF-α (**c**) and IL-1β (**d**). **e** Western blot analysis for the protein expression of TNF-α and IL-1β. GAPDH was used as loading control. The relative expressions were normalized to control (**f**). Data are presented as mean ± SD. *p < 0.05, **p < 0.01, ***p < 0.001 between the indicated groups

## Discussion

In present study, we found that mechanical stretching stress stimulation induced the inflammation and degeneration in NP cells, and these effects was reversed by inhibiting NF-κB through knocking down p65 by siRNA transfection. We demonstrated that mechanical stretching stress reduced the cell viability and promoted apoptosis of NP cells, promoted NF-κB, TNF-α, IL-1β, MMP-3 and MMP13 expression, and inhibited aggrecan and collagen II expression. Inhibition of NF-κB p65 by siRNA transfection inhibited NP cells apoptosis and increased cell viability. In addition, inhibition of NF-κB prevented mechanical stretching stress-induced expression of NF-κB, TNF-α, IL-1β, MMP-3 and MMP13, while promoted aggrecan and collagen II expression. These results strongly indicated that NF-κB played essential role in IVDD and targeting NF-κB could be used to treat IVDD.

IVDD is characterized with loss of disc extracellular matrix. The MMPs, the enzymes contributing to increased matrix degradation, are up-regulated in IVDD, [22]. Activation of NF-κB induced the expression of MMP-3, MMP-9, MMP-13 in NP cells [17]. MMP-3 and MMP-13 were the main collagenases to degrade type II collagen in NP. In present study, we demonstrated that mechanical stretching stress induced the expression of NF-κB, MMP-3 and MMP-9 while inhibiting NF-κB by knocking down p65 prevented the mechanical stretching stress-induced up-regulation of MMP-3 and MMP-9 in NP cells. Our findings were consistent to previous study in which NF-κB inhibitors were used [17, 23].

High levels of IL-1β and TNF-α are associated with IVDD [24]. IL-1β is one of the predominant cytokines which are highly expressed in degenerative IVD tissues and cells. IL-1β has been shown to be involved in inflammation, apoptosis, ECM degradation and oxidative stress in NP cells [25]. IL-1β promoted NF-κB activation, resulting in increased protein expression of MMP-3, MMP-9 in NP cells, and decreased the expression of aggrecan and collagen II [17]. Recently, emerging evidence proved that TNF-α can also induce MMP3, MMP-13 expression, resulting in significantly decreased expression of aggrecan and collagen II [6]. It was described that TNF-α and IL-1β-induced expression of MMPs was mediated by NF-κB signaling pathway [26] and NF-κB inhibitors suppressed upregulation of MMPs by TNF-α and IL-1β [27]. Here we also described that inhibition of NF-κB by knocking down p65 could prevent mechanical stretching stress-induced MMP3 and MMP-13 expression, suggesting targeting NF-κB could be a useful strategy to treat IVDD.

Mechanical loading was shown to cause apoptosis in IVD [28]. The loss of NP cells played critical role in the process of IVDD [29]. Increasing evidences demonstrated that TNF-α was involved in IVD cell apoptosis. Dai and colleagues reported that TNF-α treatment significantly enhanced the apoptotic rate through promoting p53 and caspase 3 expression in NP cells [7]. IL-1β was also shown to induce apoptosis of NP cells [30]. It is described that NF-κB plays important role in apoptosis during IVDD and inhibition of NF-κB block TNF-α and IL-1β-induced apoptosis in NP cells [31]. In present study, inhibition of NF-κB by siRNA significantly reduced the NP cells apoptosis after mechanical stretching stress stimulation, strongly suggesting inhibition of NF-κB could be used as a potential therapeutic strategy to treat IVDD.

## Conclusions

In summary, our data demonstrated that knocking down NF-κB by transfecting p65 siRNA in NP cells inhibited the inflammation and degeneration in NP cells after mechanical stretching stress stimulation.

## Data Availability

The raw data supporting the conclusions of this article will be made available by the authors, without undue reservation.
